# Pharmacological Approaches to Decelerate Aging: A Promising Path

**DOI:** 10.1155/2022/4201533

**Published:** 2022-07-11

**Authors:** Bahareh Hassani, Ghazal Goshtasbi, Shirin Nooraddini, Negar Firouzabadi

**Affiliations:** ^1^Department of Pharmacology & Toxicology, School of Pharmacy, Shiraz University of Medical Sciences, Shiraz, Iran; ^2^Student Research Committee, Shiraz University of Medical of Sciences, Shiraz, Iran

## Abstract

Biological aging or senescence is a course in which cellular function decreases over a period of time and is a consequence of altered signaling mechanisms that are triggered in stressed cells leading to cell damage. Aging is among the principal risk factors for many chronic illnesses such as cancer, cardiovascular disorders, and neurodegenerative diseases. Taking this into account, targeting fundamental aging mechanisms therapeutically may effectively impact numerous chronic illnesses. Selecting ideal therapeutic options in order to hinder the process of aging and decelerate the progression of age-related diseases is valuable. Along therapeutic options, life style modifications may well render the process of aging. The process of aging is affected by alteration in many cellular and signaling pathways amid which mTOR, SIRT1, and AMPK pathways are the most emphasized. Herein, we have discussed the mechanisms of aging focusing mainly on the mentioned pathways as well as the role of inflammation and autophagy in aging. Moreover, drugs and natural products with antiaging properties are discussed in detail.

## 1. Introduction

Aging is a biological course in which cellular function declines in a time-dependent manner, leading to reduced quality of life [1]. Aging is a multifaceted process in which a combination of environmental and genetic factors plays a role. Notably, the global population of people over the age of 65 is growing rapidly and is expected to reach 1.6 billion by the year 2050 [2]. Accordingly, aging is the principal risk factor for many illnesses such as cancer, cardiovascular disorders and neurodegenerative diseases like Alzheimer's disease. Therefore, most elderly are being treated for a variety of chronic diseases and are suffering from side effects of the drugs [2]. Specifically, only a 2% hindrance in the progression of aging, comparing with treatment of a disabling illness such as cancer would end up to a 10 million rise in healthier individuals and saving a large amount of budget [3]. Hence, identifying smart therapeutic options that uphold the process of aging on one hand and simultaneously cease or decelerate the progression of age-related illnesses is of great significance [4]. Considering the main hallmarks of aging, genetic damage is among the most important factors. Endogenous and exogenous causes can affect DNA integrity and stability by causing mutations and deletions in mitochondrial and nuclear DNA. Although the body has its compensatory mechanisms for dealing with these changes, nuclear defects can lead to premature aging syndrome and genome instability [5, 6].

Telomere curtailment is another hallmark which contributes to age-related deterioration and accelerated aging caused by pathological telomere dysfunction. Telomere lengths are heterogeneous in chromosomes, cells, and populations. Telomere length decreases when human cells proliferate and its length determines cellular life [5, 7].

In addition to the role of telomere curtailment in the process of aging, various epigenetic alterations happen in the process of aging as well which includes changes in DNA methylation patterns, posttranslational modification of histone, and chromatin remodeling. These changes can affect transcription, translation, stabilization, and degradation of molecular components. These processes can lead to cancer, inflammation, osteoporosis, neurodegenerative diseases, and diabetes. Consequently, they can increase morbidity and accelerate aging [5, 8].

Another common feature of aging is proteostasis which is characterized by the presence of nonnative protein aggregates in different tissues. Studies show that improving cellular proteostasis increases longevity and delays the progression of age-related diseases. Chaperons and proteolytic systems are the main players in proteostasis maintenance. These components decide the fate of the unfolded proteins [5, 9].

Regulation of nutrient-sensing mechanisms and pathways has been also linked to longevity since simple organic compounds such as glucose, lipids, and amino acids are involved in producing energy or are considered main constituents of cellular biomass. Different pathways are involved in nutrient sensing including the IGF-1, mTOR, AMPK, sirtuins, and insulin signaling pathways. Mutations and genetic disorders reduce the function of growth hormone, IGF-1 receptor, and other signaling molecules such as AKT, mTOR, and FOXO [5, 10].

Mitochondria are important organelles in nearly all eukaryotic cells that play an important role in energy metabolism as well as other cellular processes. The efficacy of the mitochondrial respiratory chain and ATP generation declines as organisms and cells grow. Oxidative stress is the cause or consequence of mitochondria dysfunction. ROS generated by mitochondria may affect many intracellular components such as mtDNA. Thus, it can accelerate aging and age-related diseases in mammals [5, 11].

Alteration in intercellular communication including neuronal, endocrine, or neuroendocrine changes can also affect the mechanical and functional characteristics of all tissues. Inflammatory cytokines and the processes involving ROS production, along with contagious aging in cell-cell contacts, are types of impaired intercellular communication that accelerate aging [5].

Cellular senescence is another important element involved in aging and age-related diseases and is defined as arresting a stable cell cycle in diploid cells and limiting their proliferative time. Cellular senescence increases cell cycle inhibitors and causes impaired tissue regeneration [5, 12].

Many cellular and signaling pathways are involved in the process of aging amid in which mTOR, SIRT1, and AMPK pathways are the most highlighted. Activation of SIRT1 and AMPK pathways along with inhibition of the mTOR pathway will cause antiaging effects. mTOR is considered the most influential mediator in extending lifespan and slowing aging down. Together with these mentioned pathways, the processes of autophagy and inflammation are also significantly crucial in the process of aging. Beside life style modifications, various drugs and natural products may render the process of aging.

In this review, we have emphasized on the mechanisms of aging, the involved signaling pathways, and the drugs and natural products with antiaging properties and discussed the possible implications for antiaging therapeutic interventions.

## 2. Factors Affecting Aging

### 2.1. Calorie Restriction (CR)

Calorie restriction (CR) is decreasing dietary intake below energy needs of the body, despite the fact that optimal nutrition is maintained. [13]. In CR, the amount of calories received is reduced by 60-90% over a period of time, but malnutrition does not occur [14]. CR can affect nutrient signaling, energy metabolism, and autophagy. Additionally, CR exhibits anti-inflammatory and protective neurovascular effects as well as reducing the metabolic rate [14, 15]. To date, CR is the only nutritional intervention which is recognized to attenuate aging [16–18]. CR slows down metabolism. People with higher metabolic rates have shorter lifespans [19, 20]. Metabolic rate is the energy consumed by a resting organism to maintain body functions such as metabolic homeostasis, heart rate, blood pressure, respiration, cell regeneration, nervous system activity, and ion gradient maintenance [21]. Metabolic dysfunction that occurs with age can be due to the accumulation of ROS that can disrupt cellular and molecular structures [5]. Thus, CR can reduce metabolic rate and as the result oxidative stress declines in cells and tissues. Ultimately CR improves metabolic health and increases longevity [18].

Following aging, changes occur in neurotransmitters and the neuromodulatory system. CR can exert its antiaging effects by regulating these changes and affecting the neuromodulatory system [22, 23]. It can also regulate peripheral hormones such as insulin and leptin and metabolic parameters such as glucose [24–26], which ultimately leads to reduction of insulin signaling. Studies in different species have shown that decreased insulin signaling leads to increased life expectancy [27–29]. When blood levels of insulin and glucose incline, glucose is absorbed by peripheral cells and is converted to ATP. As a consequence of increase in the level of ATP a direct by-product of ATP, ROS, rises. Therefore, lower levels of blood glucose and insulin will end up to lower levels of ROS produced in the cells [30]. Insulin also sends positive growth and proliferative signals, leading to cell growth and division. Following an increase in metabolism, ROS is produced in the mitochondria, and the time to repair and replace damaged or aging molecules is reduced. These rapid cell division rates can be detrimental even though there is enough energy to produce daughter cells. Therefore, CR may increase longevity by reducing cell division rates and maintaining cellular health [16].

Increased signaling of hormone/IGF-1 pathway leads to aging as well by increasing cell growth and proliferation. As the speed of cell proliferation increases, the body fails to detect all defects. CR has been shown to reduce the signaling of hormone/IGF-1 pathway and by this means alter cell growth and proliferation in order to maintain cellular repair and health [31, 32]. Since a report from a human study has found no change in circulating IGF-1 levels, it can be concluded that the effect of CR on IGF-1 may only be observed in animal models and not humans or that CR increases health span by acting on pathways other than IGF-1 [16, 31, 33].

Although the mechanisms of CR that lead to increased life span are not fully understood, the epigenetic mechanisms have recently been highlighted in this regard. Epigenetic changes ensue with aging, which can also be associated with the progression of age-related diseases. Although studies related to the function of epigenetic modifications in CR-associated longevity do not have a long history, however, by studying and clarifying the process, we can offer promising opportunities to postpone human aging and delay age-related diseases [34]. Epigenetic mechanisms can dynamically influence the regulation of gene expression. Three general types of epigenetic changes that are considered as the main regulators of the aging process include DNA methylation, histone modifications, and noncoding RNAs [5, 35–37]. DNA methylation is one of the most important epigenetic modifications. Studies have shown that CR can affect the expression of age-related genes through DNA methylation [38]. As we age, genomic DNA methylation patterns change which may lead to age-related diseases [39–41]. The relationship between the amount of DNA methylation in the gene control region and gene activation is inverse [42, 43]. The DNA methylation process is regulated by DNA methyltransferases (DNMTs) such as DNMT1, DNMT3a, and DNMT3b [44, 45]. DNA methylation regulates gene expression and maintains DNA integrity and the stability of many biological processes such as genomic imprinting, cell proliferation, and aging [46, 47]. 5-Methylcytosine is a product of DNA methylation. Aging causes significant changes in the distribution of 5-methylcytosine in the genome, which can eventually lead to a reduction in global DNA methylation [48–50]. As we age, decline in DNA methylation occurs. However, the promoter regions of many specific genes tend to change from unmethylated to methylated. This can lead to gene silencing, which may propagate tumor formation or aging-related genes [49, 51]. Hence, in general, two major changes in DNA methylation occur in the aging process which include a global decrease and a local increase in DNA methylation. These contents may indicate the essential role of age-related DNA methylation changes in the aging process [34].

Another epigenetic marker involved in the aging process is histone modification. Histones are proteins that help form the nucleosome, which is the basic structure of chromatin. Histones form octamer cores that cause DNA to be wrapped around them. Histone tails can be affected by posttranslational modifications (PTHMs) which can eventually lead to changes in chromatin structure. Among various types of histone modification, acetylation and methylation are the most prominent ones that are effective in the aging process. These modifications mostly occur in the core, the amino- and carboxyterminal tails, and rarely in globular domains. It is clear that histone modifications play a key role in most biological processes involved in DNA manipulation and expression. It has been observed that during aging, changes in the distribution and abundance of these histone modifications occur. Whether these changes are the causes or consequences of aging is still debatable, although it is widely accepted that there is a specific link between these processes [52–54]. Histone modifications can be catalyzed by specific enzymes, including sirtuins, which affect the aging process [55]. It has been observed that sirtuin activation is followed by CR and increased NAD levels. Beneficial effects on lifespan and improving CR-related longevity are exerted, though not exclusively, by epigenetic mechanisms associated with the sirtuin signaling [56–58]. SIRT1-dependent histone modifications in response to CR can be important mediators in the effects of CR on longevity, especially with the ability to regulate the expression of key genes involved in metabolic pathways. *p16INK4a* gene is a cyclin-dependent kinase inhibitor that accumulates during the aging process and can be considered as a biomarker of senescence. SIRT1 can play a role in regulating cellular senescence by regulating *p16INK4a* gene expression. Following CR, sirtuin is activated and binds directly to the gene promoter and exerts its deacetylating effect, reducing *p16INK4a* gene expression, thereby inhibiting cellular senescence and increasing cellular lifespan [59, 60].

The third type of epigenetic change that is considered as the main regulators of the aging process is the microRNAs (miRNAs). miRNAs are a broad class of small noncoding RNA molecules. miRNAs can detect base pairs within 3′-UTR in the target gene and thus regulate posttranscriptional gene expression [61]. By binding miRNAs to the target gene, it recruits the multiprotein complex RNA-induced silencing complex (RISC). The RISC can cleave the target gene [62–64]. Studies have shown that miRNAs are expressed differently during aging [65]. Different miRNAs have been identified, and studies have shown that they are regulated during mammalian aging by comparing their tissue-specific expression in mice of different ages. In addition, it has been shown that many miRNAs can play a role in controlling aging in a variety of human cell lines, and the function of some of these miRNAs in regulating cellular aging has helped elucidate the underlying mechanisms of aging [66, 67]. CR has been shown to have the ability to affect the expression of different age-dependent miRNAs in different tissues [68].

It has been shown that the use of drugs and substances that mimic the effects of CR can also create similar beneficial effects of CR in the body. These substances are called CR mimetics (CRMs). CRM compounds include metformin, rapamycin, resveratrol, spermidine, aspirin, hydroxy citric acid, berberine, quercetin, curcumin, myricetin, nicotinamide, piceatannol, and perhexiline maleate [14]. However, not all CRMs have the same effects on lifespan as CR itself. Some CRMs have fewer effects, and the effects of some CRMs are gender dependent [14]. The combination of some CRMs can have a synergistic effect on longevity, such as the combination use of rapamycin and metformin or the combination use of resveratrol and spermidine [69, 70].

### 2.2. Gut Microbiome

Development of the gut microbiome begins in infancy or even within the mother's uterus and is influenced by the mother's microorganisms or the environment. It can be said that diet is the most important factor in the growth and maintenance of gut microbiome configuration throughout life. Gut microbiome has a great impact on various aspects of human health [71]. Today, more attention has been paid to the gut microbiome, and it has been found that the gut microbiome can be effective in causing many diseases. Gut microbiome can play a role in maintaining brain function and normal brain growth. Gut microbiome regulation can be effective in treating some neurological disorders such as Alzheimer's and Parkinson's disease and Traumatic brain injury (TBI) [72].

Older individuals have a different gut microbiome than healthy adults. It is unclear whether the change in the gut microbiome that occurs with age is a cause or consequence of aging [71]. Due to the relationship between gut microbiome, nutrition, and inflammation, it has been found that using a proper diet and food interventions to diversify the gut microbiome and positively regulate it will increase longevity and promote health in old age [73]. Probiotics and prebiotics are promising candidates for developing and maintaining the gut microbiome and increasing longevity and health in the process of aging [71]. Additionally, taking certain medications can affect the gut microbiome, and microbiome-drug-host interactions should generally be considered. Metformin has a beneficial role in the development and maintenance of the gut microbiome and can therefore reduce age-related degenerative pathologies [74]. In a study on db/db mice, the effect of berberine and metformin on the gut microbiome was investigated. Metformin and berberine have shown to improve intestinal barrier structure, reduce intestinal inflammation, and modify the gut microbiome. Furthermore, the number of bacteria producing short-chain fatty acids such as *Ruminococcus*, *Coprococcus*, and *Butyricimonas* was increased after treatment with metformin and berberine and the number of opportunistic pathogens such as *Proteu*s and *Prevotella* decreased [75]. These all support the beneficial effects of certain medications such as metformin on gut microbiome which may lead to healthier aging and increased longevity.

### 2.3. Cellular Senescence

Cellular senescence is the state of constant inhibition of cell proliferation or the fundamentally irreversible growth arrest of a cell. Cellular senescence is considered an essential process contributing to physiological dysfunctions associated with aging and age-related diseases and is a pivotal biological process which underlies aging. Normal cells become senescent following oxidative stress, mitochondrial damage, etc. A senescent cell can cause tumor suppressor activation, apoptosis resistance, frequently increased protein synthesis, profound chromatin changes, and irreversible replicative arrest. Drugs that target cellular senescence can have beneficial effects in delaying aging and age-related diseases [76–78].

Senescent cells are identified by several features such as increased activity of senescence-associated *β*-galactosidase (SA-*β*-GAL) and senescence-associated secretory phenotype (SASP). SASP involves many proinflammatory cytokines, chemokines, growth factors, and proteases that have the potential to cause aging [79]. SASP produced by the senescent cells, leads to damage to the cell itself and the surrounding healthy cells [80]. As SASP is associated with accelerated aging and inflammatory conditions, substances and drugs that inhibit SASP can be effective in ameliorating the effects of aging. The mechanism of action of SASP inhibitors is through inhibition of Wnt/*β*-catenin and inhibition of Janus kinase (JAK) and also by inducing antioxidant effects. SASP inhibitors include melatonin, astaxanthin, Ganoderma lucid, equol, klotho, and ruxolitinib.

Apoptosis is induced in senescent cells by substances called senolytics. By triggering and killing senescent cells, senolytics delay the process of aging. Senolytics exert their effects through three different mechanisms. They inhibit the Bcl-2 family and the PI3K/AKT pathway and regulate FOXO. Senolytic compounds include navitoclax, panobinostat, catechins, dasatinib, quercetin, and fisetin [81].

## 3. Signaling Pathways Involved in Aging

Sirtuin1 (SIRT1-silent mating type information regulation 2 homolog), mechanistic target of rapamycin or mammalian target of rapamycin (mTOR), and Adenosine monophosphate-activated protein kinase (AMPK) are the main pathways that affect aging. SIRT1, mTOR, and AMPK are not only affected by exercise, CR, various drugs, etc., but are also regulated by each other. By activating SIRT1 and the AMPK pathways and inhibiting the mTOR pathway, antiaging effects can be observed. AMPK and SIRT1 activate each other and inhibit mTOR. On the other hand, mTOR activates AMPK and SIRT1 [82–84]. AMPK can activate SIRT1 following an increase in NAD^+^ levels [85]. AMPK also inhibits mTORC1 both directly and indirectly. AMPK can inhibit mTORC1 directly and by phosphorylating the raptor. By activating Tuberous Sclerosis Complex 2 (TSC2), AMPK eventually causes inhibition of mTORC1 [86]. Activation of SIRT1 leads to deacetylation of liver kinase B)LKB1) and ultimately leads to activation of AMPK [85]. Although many parts of the connection between SIRT1 and mTOR are not yet fully understood, it is known that SIRT1 can inhibit mTOR by acting on TSC2 [87]. The three main mentioned pathways involved in the aging process are depicted in Figure 1.

### 3.1. mTOR Signaling Pathway

mTOR is a serine/threonine protein kinase a member of the PIKK (phosphatidylinositol-kinase-related kinases) family that is produced by two different protein complexes, mTORC1 and mTORC2 [88]. The two complexes are different in structure and function.

The protein components of mTORC1 include the following:

1. mTOR and regulatory-associated protein of TOR (raptor)
2. Mammalian lethal with sec-13 protein 8 (mLST8)
3. Proline-rich Akt substrate 40 kDa (PRAS40)
4. DEP-domain containing mTOR-interacting protein (DEPTOR) [89].

mTOR, raptor, and mLST8 are core components of mTORC1. PRAS40 and DEPTOR are inhibitory subunits of mTORC1 [90].

The protein components of mTORC2 include the following:

1. mTOR and stress-activated protein kinase-interacting protein 1 (mSIN1)
2. Rapamycin insensitive companion of mTOR (Rictor)
3. Protein observed with Rictor 1 and 2 (protor1/2)
4. DEP-domain containing mTOR-interacting protein (DEPTOR)
5. Mammalian lethal with sec-13 protein 8 (mLST8) [89].

Protein synthesis can be controlled by mTORC1. mTORC1 has translational control by phosphorylating translation regulators eukaryotic initiation factor 4E (eIF4E) binding protein 1 (4E-BP1) [91, 92] and ribosomal protein S6 kinase 1 (S6K1) [92]. A study that was performed *in vivo* showed that homozygous mutation in ribosomal S6 protein kinase 1 (S6K1) increases lifespan [93]. mTOR can also be involved in the regulation of autophagy via the Unc-51-Like Autophagy Activating Kinase 1 (ULK1) pathway [94].

mTORC2 has the ability to control several members of the AGC kinase subfamily downstream of its pathway. These AGC kinases include Akt/protein kinase B (PKB), serum- and glucocorticoid-induced protein kinase 1 (SGK1), and protein kinase C-*α* (PKC-*α*). mTORC2 regulates survival/metabolism of cells as well as regulating cell shape by affecting the actin cytoskeleton. Cell survival effect of mTORC2 is due to its ability to activate Akt and SGK1 [89, 95]. mTORC2 can also regulate actin cytoskeleton organization. This function occurs through the activation of PKC-*α*, paxillin, and small GTPases, Rho and Rac [89]. mTORC2 induces phosphorylation and regulation of Akt/PKB. Rictor, as a protein component of mTORC2, directly phosphorylates Akt. Akt is involved in cellular processes such as apoptosis, survival, growth, proliferation, and metabolism [96]. mTORC2 can directly activate SGK1. SGK1 is a kinase that controls ion transport and growth. SGK1 is activated by mTORC2 and controls FoxO1/3a phosphorylation, ultimately leading to cell survival and cell proliferation [97, 98, 89].

Influencing factors in the upstream of mTOR that control mTORC1 function include intracellular and extracellular signals [99]. Factors affecting mTORC1 function include oxygen, ATP, amino acids, metabolic intermediates, glucose, energy, stress, hormones, and growth factors (such as insulin/IGF1) [90, 100, 99]. mTORC2 is more affected by growth factors and insulin/PI3K signaling [90]. Upstream of mTORC1 is the AKT/TSC1/2 pathway. TSC2 negatively regulates mTORC1, and Rheb binding to GTP is required for mTORC1 functionality [101]. mTORC1 plays a key role in regulating protein, lipid, and nucleotide synthesis. It also controls the process of autophagy. Thus, mTORC1 balances anabolism and catabolism under the influence of environmental factors and intracellular and extracellular signals [90]. In addition to biosynthesis pathways and autophagy, mTOR pathways have regulatory roles in mRNA translation, endoplasmic reticulum stress, mitochondrial function, cell stem regulation, and immune and stress responses. Therefore, mTOR pathways are influential in many aging-related processes [100, 102].

Additionally, longevity-dependent phenotypic features may be related to mTOR signaling pathways. Differences in gene expression and mTOR protein content are related to species longevity. In long-lived animals, *mtor* gene expression is decreased but *Raptor* gene expression is increased. There is also a difference in the protein content of mTOR in long-lived animals. As the mTOR protein content decreases, the Raptor protein declines and PRAS40 is increased. In long lived animals, it has been observed that phosphorylation of mTOR^Ser2448^/mTOR protein increases and PRAS40^Thr246^/PRAS40 decreases. There is a negative association between protein content of mTOR and PRAS40 with degree of phosphorylation. Arginine and methionine and metabolites of methionine (SAM and homocysteine) are mTOR activators; therefore, they have a negative relationship with longevity. Moreover, FKBP12 (*fkbp1a* gene expression) which is a receptor for immunosuppressant drugs like rapamycin as a regulatory factor has negative relationship with longevity [102].

### 3.2. Sirtuin Signaling Pathway

Sirtuins are nicotinamide dinucleotide- (NAD+-) dependent deacylases. There are seven mammalian sirtuins, SIRT1–7. Sirtuins have different subcellular localizations. SIRT1 is mostly nuclear; however, some of its isomers have also been detected in the cytoplasm [103]. SIRT1 is able to regulate the metabolic pathway and cellular senescence, cell survival, circadian rhythms, controlling gene expression, endothelial functions, and inflammation [104]. SIRT1 works by deacetylating the lysine groups in proteins. These proteins can be histone or nonhistone, such as transcription factors that include FOXO, p53, PGC-1*α*, MyoD, FOXO, NF-*κ*B, and Nrf2 [105]. SIRT1 plays a major role in regulating cellular senescence, and when activated, it ultimately causes antiaging effects. In general, SIRT1 exerts its antiaging effects by affecting various parts of the cellular process, such as mitochondria homeostasis, metabolism, autophagy, apoptosis, DNA repair, and the regulation of oxidative stress [106].

### 3.3. AMPK Signaling Pathway

AMPK is a complex consisting of *α*, *β*, and Ƴ subunits. *α* is a catalytic subunit, and *β* and Ƴ are regulatory subunits. AMPK is activated by phosphorylation of threonine 172 in the amino-terminal kinase domain of the *α*-subunit [107]. AMPK is a highly protected sensor that is sensitive to increasing AMP and ADP levels [108]. It is activated when the cellular energy level is low. AMPK affects many physiological processes and ultimately leads to increased energy production and reduced ATP usage [107]. AMPK has a regulation site for both ATP and AMP. The presence of AMP and ATP leads to activation and inhibition of AMPK, respectively [109]. Factors such as glucose deprivation and CR can increase the AMP to ATP ratio by reducing ATP production and ultimately leading to AMPK activation. On the other hand, exercise also increases AMP to ATP ratio by increasing ATP consumption thus activating AMPK [110]. Upstream molecules of AMPK include Ca^2+^/calmodulin-dependent protein kinase kinase *β* (CaMKK*β*), liver kinase B1 (LKB1), and transforming growth factor-*β*-activated kinase 1 (TAK1) that can phosphorylate and activate AMPK [111]. Increased ROS production as well as increased intracellular Ca^2+^ levels as a consequence of inflammatory stimuli can lead to increased CaMKK*β* activity. LKB1 expression increases via an increase in AMP to ATP ratio [112, 113]. Upstream of the AMPK pathway also includes phosphatases such as protein phosphatase 2A (PP2A) and protein phosphatase 2C (PP2C), which avert persistent activation of AMPK by dephosphorylating AMPK [114, 115]. Additionally, the downstream pathways of AMPK include SIRT1, TSC1/2, p53, GLUT1/GLUT4, ACC1, SREBP1, ULK1, and HuR.

AMPK has antiaging effects through various mechanisms. It regulates autophagy and reduces inflammation and oxidative stress. As a consequence of phosphorylation and activation of ULK1 via AMPK, the autophagy cascade initiates. Therefore, one of the mechanisms by which AMPK affects autophagy is by directly activating ULK1. AMPK can also indirectly affect ULK1 and autophagy by inhibiting mTORC1 and blocking its inhibitory effect on ULK1 [116, 117, 110]. AMPK also activates SIRT1, so it can exert its antiaging role by affecting FOXO, PGC1*α*, p53, NF-*κ*B, and Nrf2 indirectly [108].

Human antigen R (HuR) is involved in regulating the expression of genes whose expression decreases during senescence. Increased HuR expression in senescent cells leads to the maintenance of the “young cell” phenotype. Decrease in HuR expression also highlights the senescent phenotype. It has been shown that AMPK can lead to premature senescence by suppressing RNA-binding protein HuR. In general, AMPK probably plays a negative role in the aging process via this mechanism [118, 111].

AMPK inhibits mTOR by affecting TSC1/2, so it can also exert its antiaging effects indirectly via this pathway [86]. AMPK is able to activate p53, leading to restriction of cell proliferation. p53 usually inhibits cell transfer from G1 to S phase. There is a point of view that when cell proliferation is restricted, mutation accumulation does not occur in the cells and malignancy is prevented [119, 120]. AMPK can phosphorylate thioredoxin-interacting protein (TXNIP) and TBC domain family member 1 (TBC1D1) thus, translocating GLUT1 and GLUT4 [121]. Therefore, activation of AMPK can lead to increased GLUT4 and GLUT1 translocation and ultimately increasing glucose uptake [111]. Acetyl-CoA carboxylase 1 (ACC1) is a rate-limiting enzyme in the synthesis of fatty acids. It can convert acetyl-CoA to malonyl-CoA. AMPK can inactivate ACC1 by direct phosphorylation. Therefore, AMPK also plays a role in controlling cellular lipid metabolism by inhibiting ACC1 [110, 122]. Sterol regulatory element binding protein 1 (SREBP1) is a transcriptional regulator for lipid synthesis. AMPK can inhibit SREBP1 by phosphorylation. Therefore, AMPK inhibits transcription of lipogenic enzymes by inhibiting SREBP1 [123].

Figure 2 depicts an overview of the upstream and downstream of AMPK pathway.

## 4. Drugs with Antiaging Properties

### 4.1. Rapamycin

Rapamycin was first identified as an antifungal metabolite [124] and was found in a bacterium (Streptomyces hygroscopicus) that inhabited in the Easter Island (Rapa Nui) soil [124]. Immunosuppressive, antiproliferative, and anticancer properties of rapamycin was later on discovered [125]. The Food and Drug Administration (FDA) approved rapamycin as the first pharmacological agent that influences longevity in the mammalian species [126].

As said previously, mTOR plays a substantial role in aging and longevity. The role of mTOR signaling pathway in longevity and extend of life span has been studied in *Caenorhabditis elegans* [127, 128], *Drosophila melanogaster* [129], *Saccharomyces cerevisiae* [130, 131], and mice [132–135] [136]. In general, inhibition of the mTOR pathway, either genetically or pharmacologically, has shown to increase lifespan in different species [137]. The antiaging effects of rapamycin are exerted through various mechanisms, but the main route of action of rapamycin on the aging process is through inhibition of mTOR pathway. As mentioned, activation of SIRT1 and AMPK occurs following inhibition of mTOR, so rapamycin can also be indirectly effective in the aging process by activating SIRT1 and AMPK following inhibition of the mTOR pathway [82, 84, 138]. Regarding the inhibition of mTOR pathway, rapamycin inhibits both mTORC1 and mTORC2. However, its effect on mTORC2 is more complex. mTORC2 is rapamycin-insensitive. Rapamycin can inhibit mTORC2 indirectly and under prolonged exposure [139, 140]. Rapamycin binds to the cyclophilin FKBP12 and creates FKBP12-rapamycin complex. FKBP12-rapamycin complex interacts with FRB domain (FKBP12-rapamycin binding domain) of mTOR and ultimately inhibits mTORC1 activity [141, 142]. ULK1, elf4E, and S6K are downstream molecules of the mTORC1 pathway that regulate protein and nucleotide synthesis, as well as autophagy [91–94]. AKT and SKG1 are located downstream of the mTORC2 pathway, which are involved in cell survival, cell proliferation, and metabolism [89].  Figure 3 depicts antiaging mechanisms of rapamycin.

Mutation in mTOR or FKBP12 leads to rapamycin insensitivity, since it reduces the ability of rapamycin to bind to its target. Defects or mutations in mTOR-regulator proteins such as 4E-BP, S6K1, P27 ^Kip1^, and PP2A-related phosphatases may also cause rapamycin resistance. Other influential factors in rapamycin resistance include the status of p53, ataxia telangiectasia mutated (ATM), and PTEN/AKT (phosphatase and tensin homolog/protein kinase B) [143].

Rapamycin exerts its antiaging properties in the following manners:

1. Prolonging lifespan and slowing down aging.
2. Prolonging lifespan by influencing nonaging factors such as metabolic diseases and fatal neoplastic diseases [144]

Studies in different species have shown that rapamycin is also effective in a wide range of age-related conditions such as immunosenescence, age-related neurodegeneration, Alzheimer's disease, Huntington's disease, and Parkinson's disease, age-related macular degeneration (AMD), musculoskeletal disorders, cardiovascular diseases (CVDs), and age-related cancers [145]. An important characteristic of rapamycin is its anticancer properties which may also affect longevity [146–149].

Functions of many organs and associated systems are affected during aging. The immune system function decreases as a matter of aging. In this regard, on one hand the body's ability for clearing senescent cell decreases, and on the other hand, it does not have its former ability to fight infections. As known, mortality rate from infectious diseases is higher in older ages, which may be due to reduced immune function in old ages. One of the mechanisms by which the immune system is rejuvenated is the activation of autophagy. Inhibition of mTOR pathway can increase autophagy and therefore may be effective in increasing immune function during the aging process [145, 150, 151].

Regarding the effect of mTOR pathway on CNS function, it is documented that hyperactivation of mTOR is associated with brain dysfunction and cognitive deficit. mTORC1 has precise control over protein synthesis and degradation through the ULK1, S6K, and 4EBP1 pathways. The mTOR pathway also influences the progression of neuronal degradation by regulating inflammatory responses [152, 153, 145]. A study has shown that lifelong rapamycin administration in mice prevents age-related cognitive decline, which may be due to suppression of IL1-*β*. Neurological diseases that can be good candidates for treatment with mTOR inhibitors include neurodegenerative diseases such as Alzheimer's disease, Parkinson's disease, and Huntington's disease with the hallmark of abnormal protein accumulation.

Old age is linked to CVDs, and the incidence of CVDs increases with age. Studies in mice have shown that rapamycin can have beneficial effects on CVDs [145]. Rapamycin can slow or reverse the progression of age-related hypertrophy, as well as improve the ventricular function of the aging heart [154]. Rapamycin exerts its cardioprotective effects by reducing pressure overload-induced cardiac hypertrophy [155] which can also lead to suppression of experimental aortic aneurysm growth [156]. Rapamycin also appears to reduce age-related inflammation in the heart [157]. All together supports the beneficial effects of rapamycin on the cardiovascular system and related CVDs.

Although rapamycin is an FDA-approved drug which possesses antiproliferative characteristics, due to its immunosuppressive properties, it may cause serious side effects. Thus, its safety of long-term use is still questionable, and its widespread application is limited. In this regard, other pharmacological compounds that act as mTOR inhibitors with less side effects may provide advantages over rapamycin and are discussed thoroughly in the upcoming sections.

### 4.2. Resveratrol

Resveratrol (trans-3,4′,5, trihydroxystilbene) is a stilbene found profoundly in peanuts, grapes, bilberries, blueberries, and cranberries. Resveratrol belongs to the polyphenol family exerting medical properties [158]. It has been suggested that eating foods rich in polyphenols may have the ability to prevent certain diseases. Resveratrol has been effective in a majority of illnesses including CVDs, diabetes, neurological disorders, cancer, and aging [159]. Studies have shown that resveratrol has beneficial effects on longevity *in Drosophila melanogaster* [160], *Caenorhabditis elegans* [160], *Saccharomyces cerevisiae* [161], *Nothobranchius furzeri* [162], and Honey bees [163]. Many studies have also been performed on mice, rats, and human cells [164].

The antiaging effect of resveratrol can be both by postponing aging and by delaying the onset of age-related diseases [165].

Like many other illnesses, neurodegenerative diseases are affected by age. Hallmarks of aging that affect neurodegeneration include mitochondrial dysfunction, cellular senescence, stem cell exhaustion, genomic instability, telomere attrition, epigenetic alterations, loss of proteostasis, and deregulated nutrient sensing [166]. Disorders such as memory loss or cognitive impairments that occur following aging can be due to oxidative stress, inflammation, and apoptosis in neurons as well as dysregulation in autophagy [167, 166]. The antiaging effect of resveratrol in neurodegenerative diseases is due to its neuroprotective effects and by means of reducing inflammation and oxidative stress in neurons, as well as increasing neurogenesis and secretion of neurotransmitters [164].

Among the age-related diseases, CVDs are remarkably frequent. The protective role of resveratrol on CVDs has been reported. Consumption of red wine which is rich in resveratrol has been reported to reduce the incidence of CVDs [168]. Resveratrol encompasses its cardioprotective effects by regulating the renin-angiotensin system (RAS) and increasing nitric oxide (NO) production, as well as reducing oxidative stress [164].

Cancer is among the illnesses which is highly affected by age. Various studies have examined the effect of resveratrol on different cancers such as colon cancer [169], ovarian cancer [170], gastric cancer [171] and prostate cancer [172],. Resveratrol induces its antineoplastic properties by inducing apoptosis and preventing cell proliferation. Resveratrol also prevents metastasis and inhibits cell migration [164].

The antiaging effect of resveratrol is exerted through several mechanisms. Resveratrol mimics the effects of CR and shows positive effects of CR in the aging process [51]. It can have antiaging effects by inducing inhibitory effects on inflammation, improving mitochondrial function, suppressing oxidative stress, and regulating apoptosis [164]. Another antiaging mechanism of resveratrol is through the activation of SIRT1. Activation of SIRT1 regulates gene transcription of peroxisome proliferator-activated receptor-*γ* (PPAR-*γ*) coactivator-1*α* (PGC-1*α*). It therefore increases the antioxidant capacity of tissues and improves mitochondrial function [173, 174]. As dysfunction of mitochondria leads to apoptosis, SIRT1 prevents apoptosis by improving mitochondrial function [175]. SIRT1 has also antioxidant effects following increased expression of glutathione peroxidase (GSH-PX) and superoxide dismutase (SOD) [175], which lead to antiaging effects. SIRT1 regulates PGC-1*α* activity and subsequently regulates some downstream transcription factors, including estrogen-related receptor (ERR), PPAR, mitochondrial transcription factor A (Tfam), and nuclear respiratory factor (NRFs) and therefore controls fatty acid oxidation and mitochondrial function [176, 177]. Moreover, SIRT1 counteracts oxidative stress by deacetylating FOXO. Following deacetylation of FOXO, the expression of catalase (CAT) and manganese superoxide dismutase (MnSOD) increases. As a result, it counteracts oxidative stress and helps DNA repair. FOXO reduces oxidative stress damage in another way as well. Following deacetylation, FOXO is degraded (by Ubiquitination) so it loses its ability to induce cell death. By this means, FOXO regulates apoptosis and inhibits oxidative stress and cell proliferation [178, 179]. SIRT1 also controls apoptosis and oxidative stress by inhibiting p53. SIRT1 deacetylates p53, which in turn increases MnSOD expression. Eventually, the antioxidant capacity increases and regulates cellular apoptosis. In general, p53 controls the expression of many genes and can play a role in differentiation, apoptosis, regulation of metabolism, induction of senescence, and increase in cell survival [180]. SIRT1 can also play a role in longevity by inhibiting NF-*κ*B signaling pathway and in two different ways [181]: first by inhibiting inflammation and second by controlling apoptosis. In general, NF-*κ*B plays an important role in inflammatory responses. SIRT1 directly targets the p65 subunit in NF-*κ*B and regulates the expression of inflammatory factors such as IL-1, IL-6, IL-8, and TNF-*α* [182, 181]. Thus, SIRT1 is involved in the process of aging by inhibiting inflammation. NF-*κ*B can control apoptosis by regulating the expression of Bcl-2 family, TNFR-associated factor (TRAF1, TRAF-2) genes, and the inhibitor of apoptosis proteins (IAPs) which are all categorized as antiapoptosis-related genes [183, 182]. Another mechanism by which SIRT1 applies its role on aging is by stimulating Nrf2. Nrf2 is a transcription factor that increases the expression of its downstream genes, which leads to increased activity of antioxidant enzymes such as SOD and CAT [164] which can eventually inhibit ROS production. Thus, oxidative stress is inhibited, and antioxidant effects are observed [184]. Nrf2 can also have anti-inflammatory effects by reducing the activity of inflammatory cytokines such as IL-1 and TNF-*α* [185]. Hence, in general, it can be said that the antiaging effects caused by Nrf2 seek to inhibit oxidative stress and inhibit inflammation [164].

Another target of resveratrol is AMPK [182]. AMPK can be activated by metformin and resveratrol as well as in the conditions such as lack of energy and CR [108]. Activation of AMPK by resveratrol occurs when intracellular calcium levels increase [186]. SIRT1 and AMPK can stimulate each other and affect each other's activity. AMPK can activate SIRT1 following an increase in NAD^+^ levels. As said, NAD^+^ is considered a cofactor in SIRT1 activity [85]. On the other hand, AMPK reduces oxidative stress and prevents proliferative dysfunction by activating FOXO [187]. AMPK prevents aging by affecting FOXO, PGC1*α*, p53, NF-*κ*B, and Nrf2. In general, following the activation of AMPK, oxidative stress decreases, autophagy increases, and inflammation is inhibited. Thus, AMPK affects aging through various mechanisms [108].

Resveratrol can also exert its antiaging effects by inhibiting mTOR. Resveratrol can increase the expression of Rictor, a component of mTORC2, thereby activating Akt pathway and inducing autophagy. It can also eventually inhibit mTORC1 [188]. Resveratrol can also activate the PI3K/Akt/mTOR pathway, thereby inducing apoptosis [189]. The effects of resveratrol on mTOR can vary at different doses. Low doses of resveratrol can inhibit mTOR phosphorylation in serine 2448, but high doses of it can increase mTOR phosphorylation in serine 2481 [188].

Mechanistic effects of resveratrol on longevity are depicted in Figure 4.

### 4.3. Metformin

Metformin (1,1-dimethyl biguanide) is a biguanide and an FDA-approved antidiabetic for the first-line treatment of type 2 diabetes. Metformin is derived from *Galega officinalis* and has a natural base. Metformin can lower plasma glucose levels and reduce the amount of glucose absorbed by the body and the amount of glucose produced by the liver. Metformin also enhances tissue sensitivity to insulin [190]. The substantial role of metformin by numerous mechanisms in various illnesses has been reported [191–193]. The effect of metformin on life span has been documented in *C. elegans* (cocultured *with Escherichia coli*) [194–196], mice [197–199], and human [200, 201]. However, in studies performed on rat [202] and *Drosophila melanogaster* [203], no effect regarding the increase of lifespan was observed with metformin [203].

The protective role of metformin in reducing the risk of CVDs, dementia, cancer, and neurodegenerative diseases has repeatedly been reported. However, studies on longevity and mechanisms of aging have been proposed in recent decades. So human aging can be targeted while avoiding many age-related consequences at the same time.

Antiaging effects of metformin are governed by several mechanisms. In general, metformin activates AMPK [204, 205] and inhibits mTOR [206], downregulates IGF-1 signaling, reduces insulin levels [207], and inhibits electron transport chain (ETC) and mitochondrial complex 1 [208].

Cellular uptake of metformin happens via organic cation transporter 1 (OCT1). Metformin inhibits mitochondrial complex 1 in the ETC, which in turn leads to the antiaging effects of metformin by two mechanisms, AMPK-dependent and AMPK-independent [209, 210]. In AMPK-independent pathway, following the reduction of ROS and advanced glycation end products (AGEs), DNA damage is reduced and oxidative stress is inhibited [209]. In the AMPK-dependent pathway, following inhibition of mitochondrial complex I, an increase in the AMP/ATP ratio is observed, which leads to AMPK activation [210]. ULK1, PGC-1*α*, mTOR, and SIRT1 are present in the downstream of AMPK, which can be effective in the aging process [211]. Activation of PGC-1*α* increases antioxidant capacity and mitochondrial biogenesis [174]. Autophagy is induced following the activation of the ULK1 pathway [212]. As a consequence of AMPK activation, mTOR is inhibited and SIRT1 is activated. p53, FOXO, and NF-*κ*B as the downstream molecules of SIRT1 are the among the main players in longevity [212]. Following inhibition of the p53 pathway, oxidative stress is reduced and apoptosis is regulated [180]. Additionally, inhibition of NF-*κ*B also inhibits inflammation and apoptosis [181]. FOXO has beneficial effects on the aging process by regulating apoptosis and creating stress defense [179]. The effect of AMPK on mTOR is through TSC2. Downstream molecules of mTORC1 are elf4E and S6K, which play substantial antiaging by regulating translation and transcription. Protein synthesis is regulated by elf4E and S6K. S6K is also involved in the synthesis of nucleic acids [91]. Another antiaging mechanism applied by mTOR is via the ULK1 pathway. mTOR is involved in the regulation of autophagy through the ULK1 pathway [94]. Other mechanisms involved in the antiaging properties of metformin include Nrf2/glutathione peroxidase 7 (GPx7), which reduces stem cell exhaustion and inflammation. Metformin exerts its antiaging effects by acting on the Nrf2/GPx7 pathway, which increases GPx7 expression. GPx7 is an antioxidant enzyme whose expression is stimulated by Nrf2. As cells age, a decrease in the expression of Nrf2 and GPx7 is observed, which causes the accumulation of markers of oxidative stress [213].

Metformin also inhibits inflammation and reduces inflammatory cytokines by inhibiting the NF-*κ*B signaling pathway [209]. Another anti-inflammatory mechanism of metformin is by reducing inflammatory cytokines and increasing noninflammatory cytokines. Metformin can decrease TNF*α*, IL-6, and IL-1, which are inflammatory cytokines, and increase IL-10 and IL-4, which are anti-inflammatory cytokines [214]. It has been found that the level of proinflammatory cytokines such as TNF-*α* and IL-6 and the level of acute phase proteins such as serum amyloid A (SAA) and C-reactive protein (CRP) have been doubled or quadrupled in the elderly compared to the young [215]. That is suggestive of the role of aging in the rise of these markers. Inflammatory cytokines play a role in diseases that develop in old age. High levels of IL-6 are known to be a risk factor for thromboembolic complications. TNF-*α* has also been shown to play a role in Alzheimer's disease, diabetes, and atherosclerosis [216]. There are probably several mechanisms involved in age-related inflammation. Many of the factors that are responsible for the up rise in the age-related inflammation are associated with age. There is a potential decrease in the function of the immune system, which leads to an increase in inflammatory conditions. The prevalence of inflammatory diseases also increases with age. As aging happens, oxidative stress, which plays an influential role in causing inflammation, increases. ROS activates toll-like receptors (TLRs) on immune cells, which eventually leads to the activation of the inflammatory cascade [217]. Metformin can increase thioredoxin reductase (TrxR) expression in the AMPK-FOXO3 pathway, thereby reducing the intracellular amount of ROS [218].

Another antiaging mechanism of metformin is through inhibition of insulin/IGF1 signaling pathway. Following downregulation in insulin/IGF1 signaling, protein synthesis and apoptosis are regulated, and oxidative stress is inhibited. Inhibition of insulin/IGF1 signaling leads to inhibition of mTORC1 [209, 219]. Factors that reduce insulin/IGF1 signaling, such as CR and metformin, have been shown to increase lifespan and delay the onset of age-related diseases [220].

The antiaging effect of metformin is related to changes in protein synthesis in mitochondria and intrinsic mitochondrial function [221]. High doses of metformin severely damage mitochondrial function and worsens mitochondrial function, so not only antiaging properties is not observed but it may also lead to cell damage [203]. Metformin in low doses causes mild damage to mitochondrial function. Therefore, the energy level decreases and AMPK is activated. On the other hand, an adaptive hormonal response is created, which increases the tolerance to toxic substances [222]. Therefore, the antiaging effects of metformin occurring at low doses and high doses of metformin do not have beneficial antiaging effects.

In sum, metformin affects longevity by controlling protein and nucleic acid synthesis, inhibiting inflammation, reducing oxidative stress, regulating apoptosis, controlling mitochondrial function, and reducing DNA damage.  Figure 5 shows antiaging effects of metformin on different cellular pathways.

### 4.4. Lithium

Lithium is an alkali metal that is present in trace amounts in the body [223]. Lithium is mainly used to treat bipolar disorder [224]. Lithium with its autophagy regulation mechanism is used in various diseases such as Alzheimer's, Huntington's, Parkinson's, and Prion's diseases [225] and has shown a significant role in reduction of mortality rate than other drugs used in bipolar disorder [226]. The antiaging effect of lithium may be related to autophagy regulation, increasing telomere length, and enhancement of mitochondrial function in the brain [227]. Inositol monophosphatase (IMPase) and glycogen synthase kinase-3(GSK-3) contribute to the role of lithium in the regulation of autophagy. Phosphorylation on serine 9 residue of glycogen synthase kinase-3*β* inhibits its activity. Following its inhibition, the level of Bif-1 increases and autophagy is induced. GSK-3*β* upregulates AMPK, and AMPK also affects GSK-3*β*. GSK-3*β* activates TIP60 (HIV-Tat interactive protein) and ULK1 under special serum deprivation conditions. The ULK1 complex affects Amber1, Beclin1, Bakor, Vps15, and Vps34 and induces autophagy. Lithium also inhibits IMPase and causes inositol and inositol-1,4,5-triphosphate depletion. Increased inositol inhibits autophagy so lithium with reverse function can induce autophagy [225].

Telomeres protect base pairs during cellular division. Aging causes shortening of telomere length until it becomes too short to divide and cellular senescence happens [228]. Lithium may increase telomere length [229, 230]. Additionally, lithium increases complex I and complex II activities in the mitochondrial respiratory chain and improves oxidative function. It may also reduce and prevent mitochondrial disorders as well [231].

Figure 6 demonstrates cellular pathways through which lithium affects autophagy and longevity.

### 4.5. Spermidine

Spermidine is a natural polyamine that is essential for cell proliferation and growth. Spermidine content is found in abundance in plant and fungal products such as legumes, vegetables, mushrooms, and whole-grain products. The antiaging mechanism of spermidine is associated with improved effects on various organs such as the liver and kidney and the immune and cardiovascular systems. Spermidine, as a polycation, binds to molecules such as DNA, RNA, and lipids, so it can play an important role in cellular functions [232]. Spermidine affects autophagy, inflammation, DNA stability, transcription, and apoptosis [233] [234]. The effect of spermidine on aging has been investigated and proven in Drosophila melanogaster, Saccharomyces cerevisiae, C. elegans, and mice [232, 235].

According to previous studies, spermidine can cause autophagy in multiple organs such as the liver, heart, and muscles. Spermidine induces autophagy by regulating the expression of autophagy-related genes such as Atg7, Atg15, and Atg11. Increased expression of elF5A and transcription factor EB (TFEB) by spermidine also induces autophagy. The process of autophagy begins with the inhibition of protein acetylation. Spermidine initiates autophagy by reducing the expression of EP300 acetyltransferase [234].

The anti-inflammatory properties of spermidine is through the reduced phosphorylation of Akt and MAPK, which occurs by inhibiting the translocation of the NF-*κ*B p65 subunit. Spermidine regulates lipid levels by interfering with the conversion of adipocytes to mature adipocytes. Its mechanism occurs through ANP32 blockade and its effect on HUR and PPA2Ac. As PP2AC activity decreases, HUR translocation occurs and HUR binds to C/EBP-*β* in the nucleus. Afterwards, PPAR-*γ* 2 and SREBP-1c are expressed. Following expression of these factors, adipocyte cells become mature, and the expression of major markers such as FAS and GLUT4 increases. Changes in the lipid profile modulate oxidative damage and membrane fluidity as well as signaling which may affect aging [232]. Spermidine may also be involved in reducing myopathy and skeletal muscle aging along with exercise through its effect on D-Gal and reduced apoptosis [236].

Antiaging mechanisms of spermidine are shown in Figure 7.

### 4.6. Pterostilbene

Pterostilbene (trans-3,5-dimethoxy-4′-hydroxystilbene) is an analogue of resveratrol from blueberries, which is obtained by both natural extraction and biosynthesis. Pterostilbene has anti-inflammatory, antioxidant, and antitumor effects [237] and can prevent skin aging [238]. One of the antiaging mechanisms of pterostilbene is due to its beneficial effects in aging-related diseases. Pterostilbene has neuroprotective and cardiovascular protective effects. Pterostilbene has also been shown to act as an anticancer agent [239]. A study in aged rats found that pterostilbene improved memory consolidation and cognitive performance [240]. The anti-inflammatory effects of pterostilbene seek to inhibit MAPK and decrease the levels of proinflammatory cytokines such as TNF-*α*, IL-1*β*, and IL-6 [241].

In a study investing the effect of pterostilbene on sepsis-induced liver injury, it was found that pterostilbene activates SIRT1, so it can also affect FOXO1, p53, and NF-*κ*B. Pterostilbene also decreases the levels of inflammatory cytokines such as TNF-*α* and IL-6, decreases myeloperoxidase (MPO) activity, and increases Bcl-2 expression. Accordingly, pterostilbene can have anti-inflammatory and antiapoptotic effects [242]. In chondrocytes, pterostilbene can activate Nrf2 and subsequently inhibit IL-1*β*, thereby reducing ROS production. It also reduces the levels of COX-2, NO, and PGE2, exerting anti-inflammatory effects and inhibiting oxidative stress [243]. Pterostilbene increases SOD and GSH and reduces ROS production through Nrf2 signaling pathway, thereby producing antioxidant effects [244]. Pterostilbene can exhibit Nrf2-dependent antioxidant responses thus preventing UVB-induced skin damage. The anticarcinogenic and antioxidant action of Pterostilbene in the skin seeks to maintain the skin's antioxidant defense and inhibit oxidative stress caused by UVB [238]. Pterostilbene suppresses LPS-induced NF-*κ*B p65 nuclear translocation, causing downregulation of IL-18, IL-6, VEGF (vascular endothelial growth factor), matrix metalloproteinases (MMP-2 and MMP-9), and NO [245]. Pterostilbene can also scavenge free radicals, thereby protecting DNA, proteins, and lipids from damage [246].

In sum, the antiaging effects of pterostilbene and the effects of pterostilbene on age-related diseases are proposed to be mediated by activating SIRT1 and Nrf2 and suppressing NF-*κ*B, reducing inflammatory cytokines and inhibiting free radicals.

Antiaging mechanism of pterostilbene is depicted in Figure 8.

### 4.7. Melatonin

Melatonin (N-acetyl-5-methoxytryptamine) is a hormone in the pineal gland that affects many physiological functions. Melatonin secretion gradually decreases with aging [247]. Melatonin secretion is also related to light intensity and is released in the dark environment; however, the secretion ceases when exposed to light [248]. Melatonin is involved in the regulation of the circadian rhythm and also exerts antioxidant effects [249]. It has been shown that maintaining the circadian rhythm or consuming melatonin can have beneficial effects on prolonging lifespan [250]. One of the antiaging mechanisms of melatonin is due to its antioxidant effects and reduction of oxidative stress, which leads to improved mitochondrial function. Melatonin has the ability to scavenge toxic free radicals and decrease ROS and can indirectly stimulate antioxidant enzymes such as GPx, glutathione reductase (GRd), and SOD [251]. Melatonin also exerts its antiaging effects by increasing SIRT1 expression [252, 253]. Activation of SIRT1 by melatonin also regulates downstream molecules involved in the aging process and age-related diseases. SIRT1 causes deacetylation in PGC-1*α*, FOXO, p53, NF-*κ*B, and Nrf2 [254, 255] and activates PGC-1*α*. PGC-1*α* can increase mitochondrial biogenesis and improve mitochondrial function [174]. PGC-1*α* can also induce antioxidant enzymes and ultimately reduce ROS production [255]. SIRT1 promotes anti-inflammatory and antioxidant effects by activating the Nrf2 pathway. Nrf2 increases the expression of antioxidant enzymes thus reducing ROS and inhibiting oxidative stress [256, 257]. Another mechanism of reduction of oxidative stress is through deacetylation of FOXO by SIRT1. FOXO can also be involved in regulation of apoptosis [179]. Melatonin also affects p53 through activation of SIRTI. SIRT1 deacetylates p53 thus inhibiting p53 activity. Following inhibition of the p53 pathway, apoptosis is induced and senescence cells are reduced [180, 258]. SIRT1 can also inhibit inflammation and reduce senescence cells by inhibiting the NF-*κ*B pathway [259].

Figure 9 demonstrates cellular pathways involved in the antiaging effects of melatonin.

### 4.8. Aspirin

Acetylsalicylic acid or aspirin is obtained from the bark of the willow tree. Aspirin has a variety of medical uses. One of the main uses is to prevent secondary CVDs. It also has analgesic and antitumor properties [260, 261]. The antiaging effects of aspirin on C. elegans, mice, and Drosophila melanogaster have been investigated [262, 263]. Lifespan increases when germ cell progenitors become ablated. One of the proposed antiaging mechanisms of aspirin is through its effect on the reduction of germline stem cells [262]. Another proposed mechanism is improving intestinal barrier function by restricting the K63-linked ubiquitination and preventing intestinal immune deficiency [264].

### 4.9. Fisetin

Fisetin (3,3′,4′,7-tetrahydroxyflavone) is a natural compound in the category of flavonoids. It is found in fruits and vegetables such as cucumber, strawberries, kiwi, apple, grape, kale, onion, and persimmon [265]. Fisetin has been shown to have antiaging and anti-inflammatory, antioxidant, anticancer, and antimicrobial effects [266, 267]. Fisetin has beneficial effects on various illnesses [268]. Fisetin can be an important molecule against several neurological diseases such as Alzheimer's, Parkinson's, and Huntington's diseases as well as schizophrenia, vascular dementia, and TBI [269]. With its anti-inflammatory effects and reduction of oxidative stress and modulation of p25, fisetin can reduce cognitive deficits and be effective in Alzheimer's disease [270, 271]. An increase in p25 levels has been observed in the brains exposed to various neurotoxic stimuli, *β*-amyloid (Ab) peptides, and oxidative stress [272]. As noted, one of the mechanisms by which Fisetin exerts its neuroprotective effects is by preventing an increase in the harmful level of p25 [269]. P25 is the proteolytic fragment of p35 that is involved in the activation of Cyclin dependent kinase 5 (Cdk5). P35 is a regulatory subunit for Cdk5. Cdk5 is a serine/threonine kinase which is involved in brain development and has the ability to phosphorylate postsynaptic or presynaptic substrates in neurons. Cdk5 activity is controlled by binding to p35 or p39 regulatory subunits. p25 has a higher diffuse subcellular distribution than p35 and also has a longer half-life [272]. In Alzheimer's disease, the regulation of the Cdk5-p35 complex in neurons is impaired and an imbalance in p25/p35 and p25 expression is increased [269].

As mentioned, Fisetin can reduce age-related decline in brain function. This action can also be due to its antioxidant and anti-inflammatory effects. Fisetin can have a direct antioxidant effect and maintain mitochondrial function in the existence of oxidative stress and increase glutathione levels in cells. It has also anti-inflammatory effects against microglial cells by inhibition of 5-lipoxygenase and decreasing the production of lipid peroxides and inflammatory products [273]. Fisetin can prevent neuroinflammation, neurodegeneration, and memory impairment by reducing oxidative stress. These functions are mediated by preventing the accumulation of ROS, inhibiting inflammatory cytokines, and regulating endogenous antioxidant mechanisms [274]. Fisetin can also reduce the effect of oxidants produced by the c-Jun N-terminal protein kinase (JNK) and NF-*κ*B signaling pathways [275, 276]. Fisetin can reduce the expression of pro-apoptotic markers such as cleaved-caspase-3, cleaved-PARP-1, and Bax in mice's brain and may also increase the expression of antiapoptotic markers such as Bcl-2 [274]. Fisetin regulates the expression of p53 and subsequently induces apoptosis. p53 is involved in apoptosis, cell cycle, and DNA repair by regulating the expression of various genes. Fisetin can also be involved in apoptosis by activating the MAPK pathway [277]. It also exhibits neuroprotective and neurotrophic effects and improve cognition by activating the Ras-ERK cascade in neurons [278, 279].

Along the neuroprotective effects, fisetin also exhibits cardioprotective properties [267]. Consumption of flavonoids such as fisetin is beneficial on vascular health and reduces the risk of CVDs such as coronary heart disease [280, 281].

Fisetin is considered as a CRMs [282]. As previously mentioned, these substances have similar effects to CR, such as reducing the risk of age-related diseases and increasing lifespan. CR regulates the pathways of intracellular signals that lead to antiaging effects [283]. It can activate SIRT1 and AMPK and inhibit mTOR [284]. By these means, fisetin can have antiaging properties and has beneficial effects in age-related diseases [282].

Fisetin has senolytic effects as well by inhibiting the PI3K/AKT pathway [285]. Downstream molecules of the mentioned pathway are involved in different parts of cellular processes by acting on the Akt/mTOR pathway [286] that eventually leads to elimination of senescent cells [287]. A study in mice found that taking fisetin reduces oxidative stress and inflammation and removes senescent cells; thus, tissue homeostasis is restored and lifespan is increased [285].

## 5. Conclusion

Aging is an unavoidable biological process characterized by progressive time-dependent deterioration of the cells and cellular function which leads to age-related diseases, decreased life span and quality of life. In other words, aging is the driving factor of numerous age-related diseases. Accordingly, some interventions may hinder and delay the process of aging; hence, it might not be an inevitable fate. Since death from age-related diseases limits longevity, a true antiaging drug must withhold or postpone age-related diseases.

Modern medicine has improved quality of life, yet in order to reach the point to hamper the process of aging, precise knowledge of the mechanisms involved will be needed. In this regard, the exact underlying mechanisms of aging stay mainly illusive to date. Various drugs with different mechanisms have been repurposed as antiaging agents although not yet approved. While a majority of these treatments have been suggested to provide beneficial effects against aging and as a consequence hindering age-related diseases, they still lack sufficient clinical data regarding their favorable effects as well as side effects especially in the elderly.

It is noteworthy that treatments for age-related diseases are effective solely in a particular illness. However, utilizing antiaging drugs by decelerating the process of aging would prevent or delay not only one specific age-related disease but may hinder age-related diseases.

Earlier therapeutic plans relied generally on affecting oxidative stress and limiting it by the use of drugs with antioxidant properties. Alongside, CR mimetics open a new venue in hindering the aging process and ameliorating age-related diseases. However, new pharmacological approaches which have been introduced to target the process of aging mainly focus on the major pathways involved in aging including activation of AMPK and SIRT1 and inhibition of the mTOR pathways, which are assumed to play pivotal roles in upholding longevity by inserting antiaging properties and not just by preventing age-related diseases.

If these repurposed drugs be approved as antiaging treatments, the advantages which will be met over the conventional drugs used to treat late-life illnesses is that by hindering the process of aging, age-related diseases will by far decease and as a consequence human health will be improved and the lifespan would be extended. Moreover, less is spent for curing such diseases and the economic burden will reduce remarkably.

This review focused on the antiaging mechanisms of different drugs as well as natural products on the process of aging in the light of hope that someday, in the near future, a smart remedy for healthy aging will be attained.

## Figures and Tables

**Figure 1:** Three main signaling pathways involved in aging. SIRT1, mTOR, and AMPK are the three main pathways influencing the aging process that are not only influenced by CR, exercise, and fasting but are also regulated by each other. AMPK and SIRT1 activate each other and inhibit mTOR. mTOR also activates AMPK and SIRT1. AMPK can activate SIRT1 following an increase in NAD ^+^ levels. AMPK can inhibit mTORC1 both directly and indirectly. AMPK can inhibit mTORC1 directly by phosphorylating the raptor and indirectly by activating TSC2.

**Figure 2:** Overview of the upstream and downstream of AMPK pathway. AMPK pathway is one of the three main pathways in the process of aging. The upstream pathways of AMPK include LKB1, CaMKK*β*, TAK1, PP2C, and PP2A, while the downstream pathways include SIRT1, TSC1/2, p53, GLUT1/GLUT4, ACC1, SREBP1, ULK1, and HuR.

**Figure 3:** Mechanistic effect of rapamycin on longevity. The antiaging effects of rapamycin are mediated by inhibition of mTORC1. Rapamycin can also inhibit mTORC2 in conditions of prolonged exposure. mTORC2 can affect mTORC1 via the AKT/TSC2/Rheb pathway. mTORC2 is involved in cell survival by affecting AKT and SKG1. mTORC2 is involved in Actin/cytoskeleton organization by affecting PKC-*α*. mTORC2 is involved in cell survival by affecting AKT. mTORC1 regulates autophagy via the ULK1 pathway. mTORC1 can regulate transcription and translation by affecting S6K; it can also regulate translation by affecting 4E-BP1.

**Figure 4:** Mechanistic effect of resveratrol on longevity. Resveratrol is involved in longevity by activating SIRT1 and AMPK. SIRT1 will deacetylate its downstream pathway, thus activating FOXO, PGC-1*α*, and Nrf2, and inhibiting P53 and NF-*κ*B.

**Figure 5:** Antiaging effects of metformin on different cellular pathways. The antiaging effects of metformin occur through several mechanisms. Metformin inhibits electron transport chain and mitochondrial complex 1 and can exert antiaging effects in the AMPK-dependent or AMPK-independent pathway. In the AMPK-independent path, it reduces ROS and AGEs. In the AMPK-dependent pathway, it activates PGC-1*α* and ULK1 and can also inhibit mTORC1. Metformin is also involved in antiaging effects by inhibiting the insulin/IGF1 signaling pathway. Other antiaging mechanisms of metformin include activating Nrf2 and inhibiting NF-*κ*B, increasing noninflammatory cytokines, and decreasing inflammatory cytokines.

**Figure 6:** Cellular pathways through which lithium affects autophagy and longevity. One of the antiaging mechanisms for lithium is autoregulation, which manifests itself through the inhibition of GSK-3*β* and IMPase.

**Figure 7:** Antiaging mechanism of spermidine. The antiaging mechanism of spermidine is associated with autophagy, inflammation, and lipid metabolism. Inhibiting the translocation of the NF-*κ*B p65 subunit reduces Akt and MAPK phosphorylation, which occurs by spermidine and reduces inflammation.

**Figure 8:** Antiaging mechanisms of pterostilbene by means of various pathways. Pterostilbene is involved in longevity with its anti-inflammatory and antioxidant effects. Pterostilbene activates SIRT1 and Nrf2 and inhibits NF-*κ*B. Following activation of SIRT1, FOXO is also activated and P53 is inhibited.

**Figure 9:** Cellular pathways involved in antiaging effects of melatonin. Melatonin exerts its antiaging effects through the activation of SIRT1 and its antioxidant effects. Following activation of SIRT1, FOXO and Nrf2 and PGC-1*α* are activated and P53 and NF-*κ*B are inhibited.

## Abbreviations

SIRT1: Sirtuin 1 = silent mating type information regulation 2 homolog
mTOR: Mammalian target of rapamycin/mechanistic target of rapamycin
AMPK: Adenosine monophosphate-activated protein kinase
IGF-1: Insulin-like growth factor 1
Nrf2: Nuclear factor erythroid 2-related factor 2
FOXO: Forkhead box protein O
NF-*κ*B: Nuclear factor kappa light chain enhancer of activated B cells
CR: Calorie restriction
CRMs: Caloric restriction mimetics
SASP: Senescence-associated secretory phenotype
Bcl: B cell lymphoma
PI3K: Phosphatidylinositol 3-kinase
AKT: Protein kinase B, PKB
JAK: Janus kinase
TSC2: Tuberous Sclerosis Complex 2
PIKK: Phosphatidylinositol-kinase-related kinases
raptor: Regulatory-associated protein of TOR
mLST8: Mammalian lethal with sec-13 protein 8
PRAS40: Proline-rich Akt substrate 40 kDa
DEPTOR: DEP-domain containing mTOR-interacting protein
mSIN1: Stress-activated protein kinase-interacting protein 1
Rictor: Rapamycin insensitive companion of mTOR
protor1/2: Protein observed with Rictor 1 and 2
FKBP12: FK506 binding protein
FRB domain: FKBP12-Rapamycin Binding domain
eIF4E: Eukaryotic initiation factor 4E
4E-BP1: Eukaryotic initiation factor 4E binding protein 1
S6K1: Ribosomal protein S6 kinase 1
ULK1: Unc-51-Like Autophagy Activating Kinase 1
PGC-1*α*: Peroxisome proliferator-activated receptor-*γ* (PPAR-*γ*) coactivator-1*α*
GSH-PX: Glutathione peroxidase
SOD: Superoxide dismutase
ERR: Estrogen-related receptor
PPAR: Peroxisome proliferator-activated receptors
Tfam: Mitochondrial transcription factor A
NRFs: Nuclear respiratory factor
MyoD: Myoblast Determination Protein 1
CAT: catalase
MnSOD: Manganese superoxide dismutase
TRAF: TNFR-associated factor
IAPs: Inhibitor of apoptosis proteins
TAME: Targeting Aging with Metformin
ETC: Electron transport chain
AGEs: Advanced glycation end products
GPx7: Glutathione peroxidase 7
TrxR: Thioredoxin reductase
MPO: Myeloperoxidase
PGE2: Prostaglandin E2
VEGF: Vascular endothelial growth factor
MMP-9: Matrix metalloproteinase-9
MMP-2: Matrix metalloproteinase-2
DPPH: 2,2-Diphenyl-1-picryl-hydrazyl
ABTS: 2,2′-Azinobis-(3-Ethylbenzothiazoline-6-Sulfonic Acid)
GPx: Glutathione peroxidase
GRd: Glutathione reductase
MAPK: Mitogen-activated protein kinase
Bax: Bcl-2-associated X protein
Caspases: Cysteine-aspartic proteases
PARP: Poly ADP- (Adenosine Diphosphate-) Ribose Polymerase
JNK: c-Jun N-terminalprotein kinase
CaMKK*β*: Ca^2+^/calmodulin-dependent protein kinase kinase *β*
LKB1: Liver kinase B1 = serine/threonine kinase 11 = STK11
TAK1: Transforming growth factor-*β*-activated kinase 1
IMPase: Inositol monophosphatase
Gsk3: Glycogen synthase kinase 3
Bif-1: BAX interacting factor 1
TIP60: Tat-Interactive Protein 60
elF5A: Eukaryotic translation initiation factor 5A
TFEB: Transcription factor EB
DNMTs: DNA methyltransferases
AMD: Age-related macular degeneration
SGK1: Serum- and glucocorticoid-induced protein kinase 1
PKC-*α*: Protein kinase C-*α*
SA-*β*-GAL: Senescence-associated *β*-galactosidase
OCT1: Organic cation transporter 1
TBI: Traumatic brain injury
Cdk5: Cyclin-dependent kinase 5
PTHMs: Posttranslational modifications
MiRNAs: MicroRNAs
RISC: RNA-induced silencing complex
SIPS: Stress-induced premature senescence
ATM: Ataxia telangiectasia mutated
PTEN: Phosphatase and tensin homolog
CVDs: Cardiovascular diseases
SAA: Serum amyloid A
CRP: C-reactive protein
TLRs: Toll-like receptors
PP2A: Protein phosphatase 2A
PP2C: Protein phosphatase 2C
GLUTs: Glucose transporters
TXNIP: Phosphorylate thioredoxin-interacting protein
TBC1D1: TBC domain family member 1
ACC1: Acetyl-CoA carboxylase 1
HuR: Human antigen R
SREBP1: Sterol regulatory element binding protein 1.
